This article has been retracted.

# Quality Assessment of Vocational Education Teaching Reform Based on Deep Learning

**DOI:** 10.1155/2022/1499420

**Published:** 2022-07-01

**Authors:** Zai Ni, Fei Wang

**Affiliations:** ^1^Dean's Office, Hangzhou Vocational and Technical College, Hangzhou Zhejiang 310018, China; ^2^Human Resources Office, Hangzhou Vocational and Technical College, Hangzhou Zhejiang 310018, China

## Abstract

In my country, vocational training is an important part of the educational system. In my country's vocational education system, there is currently a conscious focus on reform and innovation. It is critical to undertake a thorough assessment of teaching quality in vocational education in order to improve teaching quality. Artificial intelligence technology, particularly deep learning technology, can successfully handle this challenge because of the various and complicated aspects involved in the assessment of teaching quality. This article thus provides an evaluation approach for the quality of vocational education that is based on a thorough investigation. Finally, research has demonstrated that this approach is capable of objectively and fairly evaluating a teacher's teaching quality, increasing a teacher's teaching passion, improving a teacher's teaching quality, and nurturing extraordinary abilities.

## 1. Introduction

Vocational education is an educational activity implemented in order to enable learners to master professional knowledge, acquire professional skills, and form good professional ethics, so as to serve social production [1]. Therefore, vocational education is inextricably linked with the economic development of a country and a nation. With the continuous development and transformation of the economy, the connotation and types of vocational education also change and evolve. Vocational education is an important part of national education and an important source of support for social labor. Vocational colleges are the main body of vocational education, and the rational construction of the teaching system is the core of improving the quality of all schools. As the most direct way to achieve teaching goals and ensure teaching quality, the development of vocational education teaching activities is the most critical link in vocational education. Therefore, teaching innovation is the key to the successful reform of vocational education to adapt to the new economic normal and provide high-quality human capital for the new economy [2]. It was previously said by our nation's education minister that the most important job of vocational education in the future would be to increase the quality of education; this is done by enhancing teaching quality, which is done by conducting effective teaching evaluations.

The quality of vocational schools will be directly related to the development of vocational education in our country. The school's direction, educational quality, and the impact of educational reform are all determined by the quality and level of the school's teaching staff. To establish a high-quality teacher team, first of all, teachers should have a comprehensive understanding and correct evaluation. This can not only encourage teachers to improve their own quality consciousness, make them understand their own achievements and deficiencies, consciously regulate their own behavior, continuously improve and perfect their previous work, and move towards higher goals, but, at the same time, it can also promote the school leaders' awareness of the problems and importance of improving teachers' quality and teaching level enables the school to take effective measures to strengthen the construction of the teaching staff in a more targeted and planned manner. Classroom teaching is the main way for schools to achieve educational goals. From the perspective of school management, in order for school leaders and managers to have a thorough understanding of the school's teaching work and to enhance the quality of teaching, it is necessary to evaluate the quality of teachers' classroom instruction [3]. The level of teaching work has a great influence on the level of talents trained, so the evaluation of school teaching work level has become an important content of teaching management. School teaching quality assessment is a quite complicated procedure.

Teachers and students have a complicated connection in the classroom, and a variety of variables influence how well a lesson is taught. How can a scientific and acceptable teaching quality assessment system be established such that it can objectively and fairly evaluate the teaching of teachers? Quality is a very important topic. Since the birth of the concept of artificial intelligence, it has continued to develop with the transformation of computers. Artificial intelligence has mainly experienced the reasoning period in the 1960s, the knowledge period in the 1970s, and the machine learning period that started in the 1980s and continues to this day. Connectionism, statistical learning, and deep learning were the three stages of machine learning, and deep learning is currently at a stage of rapid development. Deep learning is based on neural networks for supervised or unsupervised feature learning, representation, classification, and pattern recognition through multilevel nonlinear information processing and abstraction. Unfortunately, the integration of teaching quality assessment and deep learning technology is still relatively limited. Based on this background, this paper proposes a teaching quality evaluation method for vocational education based on deep learning. Using the advantages of neural network to solve nonlinear problems, an improved method of BP algorithm and simulated annealing method is proposed [4]. On this basis, the network structure, learning parameters, and learning algorithm of the teaching quality assessment model are determined. It has realized the efficient, network, and intelligent evaluation of teaching quality [5].

The paper arrangements are as follows: Section 2 describes the related work; Section 3 defines the methods of the proposed work.  Section 4 discusses the experiment and results. In Section 5, the article comes to a close.

## 2. Related Work

Most of my country's research on vocational education reform is currently at the macro level; that is, it primarily emphasizes the importance of vocational education adapting to the new normal and reform ideas at the broadest, most specific levels. In recent years, the United States, France, Australia, Germany, and other nations have emphasized action-oriented teaching, multidisciplinary program with vocational elements, situational teaching, and “self-paced” learning in their reforms of vocational education teaching methods. For the vocational education teaching system, many countries have put the reform emphasis on the credit transfer system, the unit system, and the mutual recognition system of learning and work experience, the main purpose of which is to establish a flexible vocational education teaching system. From the 1970s to the 1980s, the German vocational education circle has attached great importance to the action orientation in teaching activities. In order to promote the more extensive and effective development of action-oriented teaching activities, Germany has implemented a series of teaching reform pilot projects related to vocational preparation education and vocational education [6]. The development of modern apprenticeship based on traditional apprenticeship is one of the important goals of British vocational education and training reform. The so-called British modern apprenticeship system can also be understood as a combination of school education and enterprise training. Finally, the comprehensive ability is improved [7].

The field of educational assessment is both old and new. It started early in the United States, Britain, Germany, and other countries. Since the end of the 19th century, it has been regarded as an independent branch subject and has gradually developed into a scientific direction. Teaching quality assessment may be accomplished via a variety of means. The commonly used evaluation methods are as follows: the existing teaching quality evaluation work is divided into two parts; one is to determine the content in the evaluation system, and the other is to classify the teaching quality according to the content score [8, 9]. It is decided what will be included in the assessment of the quality of the instruction being provided to students. It is difficult to designate a specific course, a specific learning stage, to a specific course when constructing the content of the teaching level assessment system since learning and development are ongoing processes and the learning and growing environment is various. The teacher's involvement is measured by focusing on the evaluative content of the teaching process rather than on course performance or teaching impact as the primary indication. With regard to educational processes, it is difficult to compare the teaching of different disciplines and courses of diverse type, as well as various linkages and teaching objects, because of the many factors involved. As a result, only those criteria that directly indicate the teaching level and have similar construction in the assessment system should be included. Based on the current system of evaluating teaching levels, the development of indicators is focused on the following aspects: teaching attitude, teaching material, teaching ability, teaching technique, teaching and educating people, and the teaching impact [10]. In the current teaching quality evaluation method, in order to form a total evaluation of teaching quality, it is necessary to organize students to evaluate and score the above six indicators and obtain the quality grade coefficient of each evaluation content according to a reasonable procedure and scoring method. Obviously, the grading of the total index is a classification problem. For large and complex evaluation systems, there are many evaluation indexes, the grading criteria are complex, and it is difficult to use an analytical expression to give an appropriate mathematical model, which is mostly a nonlinear classification problem [11].

Deep learning is now experiencing a surge. Neural networks are the foundation of deep learning. Artificial neural network research has gradually recovered since the 1980s, resulting in a research climax around the world. Worldwide, scientists and entrepreneurs are organizing and implementing related scientific research projects, such as the DARPA program in the United States, the HFSP program in Japan, the “Eureka” program in France, the “European Defense” program in Germany, and the “High-Tech Development” program in Russia [12, 13]. In my country, since the annual academic conference of neural network was held in 1990, artificial neural network has also become a major research hotspot in my country, and research work has been carried out in universities and research institutes. Artificial neural network is a fast-growing interdisciplinary subject, a new type of intelligent information processing system developed by learning from biological neural network. Because its structure “imitation” the biological nervous system of the human brain, it also has some kind of intelligence in function features [14]. It is similar to the method of repeated learning in the human brain, first giving a series of samples, learning, and training, so as to generate patterns that distinguish different characteristics between various samples. The sample set should be as representative as possible. In order to accurately fit various sample data, the system finally obtains potential patterns through hundreds or even thousands of training and learning times. When it encounters new sample data, the system automatically makes predictions and classifications based on the training results [15]. The unique information processing and distinctive solution capabilities of neural networks have garnered considerable interest in recent years, indicating a wide range of potential applications. For example, neural network technology has showed a remarkable ability to recognize and categorize patterns, as well as to filter out noise and anticipate future events. Unlike many older approaches, it can process almost any form of data [16]. Data that is complicated and has unknown patterns may be discovered via continual learning. The conventional analytical procedure and the challenge of picking a suitable model function form are both solved by the neural network technique. Modeling and analysis benefit greatly from the inherent nonlinearity of the process, which does not need identifying the specific nonlinear connection at hand [17]. At present, in foreign financial circles, there have been some successful examples of neural networks used in mortgage risk assessment and credit insurance analysis. These successful examples provide a new method for us to study evaluation or evaluation problems in the field of education and new ideas [18].

## 3. Method

In this section, we discuss the neural network theory, BP artificial neural network, and teaching quality evaluation model cased on neural network in depth.

### 3.1. Neural Network Theory

#### 3.1.1. Neural Network Basics

An adaptive nonlinear dynamic system is formed by a large number of neurons coupled together in an ANN. Neurons are the basic units that make up a brain network. A neuron is the smallest computational unit in a neural network. It is generally a multi-input/single-output nonlinear device. Its action is very simple. It only multiplies the input vector with the weight vector and then undergoes a transformation to obtain the output value. This output is then passed down through the interconnections of the network and becomes the input to many neurons. Neurons may be abstracted into a simple mathematical model, as illustrated in Figure 1, based on their features and functions.

In the figure, *x*_1_, *x*_2_, ⋯, *x*_*n*_ are the input of neurons; *ω*_*i*1_, *ω*_*i*2_, ⋯, *ω*_in_ are the weight coefficients of *i* neuron with *x*_1_, *x*_2_, ⋯, *x*_*n*_, respectively; *Y*_*i*_is the output of the neuron*i*; *f* is called the transfer function or the excitation function, which determines the output of the *i* neuron when the costimulation of the input *x*_1_, *x*_2_, ⋯, *x*_*n*_ reaches the threshold value. Its input-output relationship can be described as

(1) $$\begin{array}{c} I_{i}=\overset{n}{\underset{j=1}{\sum }}\omega_{ij}x_{j}-\theta_{i}. \end{array}$$

Sometimes, for the sake of convenience, *θ*_*i*_ is often regarded as the weight corresponding to the input quantity *x*_*i*0_ that is always equal to 1, which is recorded as

(2) $$\begin{array}{c} I_{i}=\overset{n}{\underset{j=1}{\sum }}\omega_{ij}x_{j}, \end{array}$$

where *ω*_*i*0_ = −*θ*_*i*_: *x*_*i*0_ = 1.

#### 3.1.2. Activation Function

The neuron should deliver the correct output after getting input from the network. Each neuron has a threshold that is based on biological neuron characteristics. When the input signal's cumulative effect exceeds a threshold value, neurons are said to be stimulated; otherwise, they should be in an inhibitory state. In order to make the system have a wider applicability, it is hoped that the artificial neuron has a more general transformation function. This is utilized to accomplish the modification of the network input that the neuron receives. Activation functions are also known as the excitation functions, and they may be expressed as either a linear or nonlinear slope function, a threshold, or S shape.

The interpretation function is also referred to as the step function. To test if the neuron's network input exceeds a predetermined threshold, the activation function is utilized. The simplest fundamental activation function is the linear function, which serves as an adequate linear amplification of the network input received by the neuron. Its general form is

(3) $$\begin{array}{c} f\left(x\right)=kx, \end{array}$$

where the magnification factor, *k*, and the displacement factor, *c*, are both constants in mathematical expressions.

*Nonlinear slope function*: the linear function is very simple, but its linearity greatly degrades the performance of the network, and it even degrades the function of a multilevel network to that of a single-level network. As a result, nonlinear activation functions in artificial neural networks are required.

(4) $$\begin{array}{c} f\left(x\right)=\left\{\begin{array}{cc} 1 & x\geq x_{0},\\ ax+b & x_{1}\leq x\leq \\ 0 & x\leq x_{0}. \end{array}\right.x_{0}, \end{array}$$

*S-shaped transfer function*: it is usually a monotonically differentiable function with continuous values in (0, 1) or (-1, 1) and is usually represented by a logarithmic or tangent type of S-shaped curve.

#### 3.1.3. Neural Networks

In an artificial neural network, a specific topological structure connects a large number of neurons in a large-scale parallel manner. A neuron is a single processing unit that is incapable of performing complex operations. Only a neural network with a vast number of neurons is capable of processing and storing complicated data and exhibiting a variety of superior properties. Therefore, the choice of connection scheme is the main problem in designing neural network systems. First and final levels of a computer's processing unit are known as “input” and “output,” respectively; additional layers are referred to as “hidden.” The number of processing units in each layer is also a matter of choice. In some networks, each processing unit of the current layer gets an input signal from the previous layer, and its output is passed to the processing unit of the next layer. Some networks allow communication between processing units between layers, and the feedback structure also needs to allow the processing units of the previous layer to accept the output of the processing units of the next layer. The feedback neural network model and the forward neural network model may be distinguished based on the architecture of the neural network. Neural network models now fall into the following categories.

There are many different types of feed-forward networks, but the most popular is the error backpropagation (BP) neural network. A multilayer mapping neural network that uses the lowest mean square error learning strategy is one of the most widely utilized neural network models presently. In addition to being the neural network model in use in this article, it is widely utilized in voice synthesis, control, recognition, and teacher training. The other neural network models are Hopfield network, Kohonen network, and neural network with radial basis function.

#### 3.1.4. Training of Artificial Neural Network

Artificial neural networks' capacity to learn is by far its most appealing characteristic. The renowned learning theorem of artificial neural networks was developed in 1962 by a group of researchers. An artificial neural network's training is the first step in the learning process. The term “training” refers to the act of adjusting the connection weights between neurons in the artificial neural network during the process of entering a sample set of sample vectors into the network. With a weight matrix, a sample set's connotation may be saved as the network takes input. It can give an appropriate output. From the perspective of advanced forms of learning, one is tutored learning and the other is tutorless learning, and the former seems to be more common. Whether students go to school to receive education from teachers or study by themselves, they all belong to tutored learning. There are still many times. People are constantly summarizing and learning through some practical experience; maybe, these should be regarded as unsupervised learning.

Learning with a mentor corresponds to training with a mentor. In this training, the user is required to give the corresponding ideal output vector at the same time as the input vector. Therefore, the network trained by this training method implements a heterogeneous mapping, and the input vector and its corresponding output vector form a “training pair.” Among the tutored training algorithms, the most important and widely used is the Delta rule. Its form is

(5) $$\begin{array}{c} \omega_{ij}\left(t+1\right)=\omega_{ij}\left(t\right)+\alpha \left(y_{i}-o_{j}\left(t\right)o_{i}\left(t\right)\right), \end{array}$$

where *ω*_*ij*_(*t* + 1) and *ω*_*ij*_(*t*) represent the weights of the connection between neurons AN_*i*_ to AN_*j*_; at time *t* + 1 and time *t*, respectively, *o*_*j*_(*t*) and *o*_*i*_(*t*) are these two neurons. The output of the unit at time *t*,*y*_*i*_, is the ideal output of the neuronAN_*j*_; *α* is the given learning rate.

### 3.2. BP Artificial Neural Network

The error backpropagation method is often used to refer to a multilayer forward neural network (BP algorithm). By reintroducing the error backpropagation method for forward neural networks in parallel distributed processing research in 1986, Rumelhart and McClelland addressed the multilayer forward neural network's learning difficulty and made it applicable in other industries. For practical applications of artificial neural networks, BP networks and their variations, which are the heart of the forward network, are widely used. This is also the most fundamental aspect of artificial neural networks. Nearly 90% of neural network applications are based on the BP algorithm, according to data.

#### 3.2.1. BP Network Structure

The BP neural network is a three- or more-layered hierarchical neural network. All three layers are included inside this structure. Because the layers are only partially interconnected, neurons in one layer are not related to those in the next. To implement the BP algorithm, a three-layer BP network with one hidden layer is shown in Figure 2.

In Figure 2, it is assumed that the number of units of the input layer, hidden layer, and output layer is *I*, *J*, and *K*, respectively; the input is (*x*_0_, *x*_1_, *x*_2_, ⋯, *x*_*i*+1_); the hidden layer output is (*h*_0_, *h*_1_, *h*_2_, ⋯, *h*_*k*−1_), the actual output of the network is (*y*_0_, *y*_1_, *y*_2_, ⋯, *y*_*k*−1_); (*d*_0_, *d*_1_, *d*_2_, ⋯, *d*_*k*−1_) represents the expected output of the training sample. The weight from the input layer unit *i* to the hidden layer unit *j* is *V*_*ij*_, and the weight from the hidden layer unit *j* to the output layer unit *k* is *W*_*ij*_ and *θ*_*i*_ and *θ*_*j*_; the hidden layer unit and the output layer unit are both represented by these symbols. Therefore, the network's hidden layer unit output is

(6) $$\begin{array}{c} h_{j}=f\left(\overset{I-1}{\underset{i=0}{\sum }}v_{ij}x_{i}-\theta_{j}\right). \end{array}$$

Each unit in the output layer has the following value as its output:

(7) $$\begin{array}{c} y_{k}=f\left(\overset{J-1}{\underset{J=0}{\sum }}w_{jk}h_{j}-\theta_{k}\right). \end{array}$$

#### 3.2.2. Learning Algorithm of Standard BP Network

Two stages are involved in the BP algorithm. First, the input sample is fed into an output layer, where it is processed by a layer-by-layer method and finally output. The weight coefficient of this process remains unchanged. Second, if the output does not match the desired output, backpropagation is entered. To reduce the deviation signal, the second stage (also known as the backpropagation process) utilizes the error calculated at each concealed layer to advance the weights of the preceding layer. The network weight adjustment adopts the Delta learning rule; that is, the gradient along the error surface descends the fastest according to the gradient method, so as to minimize the network error.

*Backpropagation stage*: the deviation signal is transferred backward according to the original forward propagation route, and each hidden layer's weight coefficient is changed to minimize the deviation signal. The ideal gradient descent technique is the most popular approach to determining the value with the lowest variance. The weight adjustment formula between the output layer and the hidden layer is shown in the following equation. The correction value for each *ω*_*jk*_ is

(8) $$\begin{array}{c} ∆\omega_{jk}=-\eta \frac{\partial E}{\partial \omega_{jk}}=-\frac{\partial E}{\partial \text{ne}{\text{t}}_{k}}∙\frac{\partial \text{ne}{\text{t}}_{k}}{\partial \omega_{jk}}=\eta \delta_{k}o_{j}. \end{array}$$

If the activation function of each layer of the BP neural network takes the unipolar sigmoid function, that is,

(9) $$\begin{array}{c} f\left(\text{net}\right)=\frac{1}{1+e^{-\text{net}}}. \end{array}$$

For the input layer,

(10) $$\begin{array}{c} ∆\omega_{jk}=\eta o_{j}\left(d_{k}-o_{k}\right)o_{k}\left(1-o_{k}\right). \end{array}$$

For the hidden layer,

(11) $$\begin{array}{c} ∆v_{jk}=\eta o_{j}\left(\left(1-o_{j}\right)\overset{K-1}{\underset{k=0}{\sum }}\delta_{k}\right.\omega_{jk}o_{i}. \end{array}$$

#### 3.2.3. Limitations and Improvement Methods of BP Network

The BP network is the most commonly utilized and has shown to be a worthwhile investment in the field. There are a slew of issues with the algorithm, though. Particularly problematic for BP's network are these five issues, some of which are quite significant. These five questions are briefly discussed below.

1. The problem of convergence speed

The biggest weakness of the BP algorithm is that its training is difficult to master. Algorithm training takes a long time, particularly after the network training has progressed to a certain point; its convergence speed may drop to a point where it is difficult to grasp, unbearable point.

(2) The BP algorithm employs the steepest descent approach to solve the local minimum point issue

The slope of the error surface is used to estimate its training. In a high-dimensional space, the error surface of a complex network may be exceedingly complicated and uneven. Many local minimums are disseminated across the network during training. With the existing approach, it is very difficult to get out of a local minimum.

(3) The problem of network paralysis

The weight may become very large during training, causing the neuron's network input to become very large, causing the derivative function of its activation function to have a tiny value at this moment. At this time, the training step length will change is very small, which in turn causes the training speed to drop very low, eventually causing the network to stop converging.

In order to overcome the problems of slow results and local minima of the BP algorithm, many scholars have revised the BP algorithm from different aspects. The following are some commonly used improved algorithms:

1. When the traditional BP method updates the weights, it does so exclusively based on the error's gradient descent direction at time *t*, which may cause the training process to oscillate and converge slowly based on the enhanced gradient descent technique. The improved technique is based on the standard gradient descent approach, which means that each time the network weights and thresholds are corrected, the previous learning's correction amount is added in a set proportion, accelerating network learning convergence
2. The BP algorithm and simulated annealing method are combined to form a new algorithm. It can not only take into account the advantages that the adjustment amount of the connection weight of the BP algorithm is determined but also take into account the randomness and heuristics of the adjustment of the connection weight in the simulated annealing algorithm. As a result, by dividing the change of a connection weight into two parts, the BP method can give the direct calculation part, while the simulated annealing approach can supply the random component [19]. The connection weight *ω*_*ij*_ between the neurons AN_*i*_ and AN_*j*_ in the network is adjusted by the following formula:

(12) $$\begin{array}{c} {\Delta \omega }_{ij}=\alpha \left(\left(1-\beta \right)\delta_{j}o_{i}+\beta \Delta \omega_{ij}^{\prime }\right)+\left(1-\alpha \right)\Delta \omega_{ij}^{\prime \prime }, \end{array}$$

where *ω*_*ij*_′ is the adjustment amount of the connection weight *ω*_*ij*_ obtained according to the simulated annealing algorithm and *ω*_*ij*_′′ is the last modification amount of *ω*_*ij*_; *α* ∈ (0, 1) is the learning rate. Here, it simultaneously also plays the role of weight distribution of “direct part” and “random part”; *β* ∈ (0, 1) is the impulse coefficient

(13) $$\begin{array}{c} \omega_{ij}^{\prime }=T\tan\left(p\left(\Delta \omega \right)\right). \end{array}$$

*p*(Δ*ω*is randomly selected in the uniform distribution interval [-0.5, 0.5];*T*is annealing temperature.

(14) $$\begin{array}{c} T=\frac{T_{0}}{1+t}, \end{array}$$

where *T* is the initial temperature and *t* is the number of annealing.

### 3.3. Teaching Quality Evaluation Model Cased on Neural Network

#### 3.3.1. Vocational School Teaching Quality Evaluation Index System

To reflect the scientificity, fairness, and rationality of teaching quality evaluation, the index system plays a key role. Different colleges and universities have different divisions of labor, positioning, and their own characteristics, and different indicators should be used for evaluation. Therefore, the establishment of a scientific and appropriate assessment index system for various colleges and institutions is necessary. The so-called scientific principle means that the established indicators and standards must reflect the development goals of education and the objective laws of teaching. Specifically, the evaluation index should be consistent with the overall goal of education and teaching; that is, whether the goal is correct or not should be measured by the correct direction. If the indicators violate the educational goals, it will lead to inaccurate goals and mistakes in decision-making and eventually lead to the wrong way of teaching. Teaching is guided by the evaluation index. A teacher's attention will be focused on what metrics are used in evaluations and assessments. Therefore, the selection and creation of indicators are critical. Reflecting the nature of education and selecting typical and objective indicators as well as paying attention to the leadership role are all necessary parts of the process. Otherwise, too simple and excessive indicators will make teaching evaluation useless.

According to the assessment index method for teaching work level in the normal colleges and universities, this paper strives to reflect the principles of scientificity, comprehensiveness, accuracy, and measurable operability and designs the index system into the following 12 indicators.  Table 1 shows the index system that defines the network structure of the model for evaluating teaching quality.

#### 3.3.2. Normalization of Input Indicators

Since the input of each indicator is obtained by students' scoring using the percentage system, the magnitude of each component's value is vastly different from the next. One possible consequence of using raw data directly is that the neuron's effective processing range may be exceeded due to the so-called “saturation phenomenon,” which occurs when an amount of raw input is applied without any treatment. Even though the total value of the original data is not excessive, the network's influence may be larger than the impact of other components because of a component's excessive size, causing other components to lose control of the network. The neural network's input samples must, therefore, be normalized. For the neural network, the input should be normalized to [0, 1]. Because sigmoid function is a linear transformation of data processing, the maximum-minimum approach is adopted in this work for normalizing because it can better keep its original meaning and will not cause information loss. In this work, the input normalization formula is as follows:

(15) $$\begin{array}{c} X=\frac{I-I_{\min}}{I_{\max}-I_{\min}}. \end{array}$$

#### 3.3.3. Evaluation Model Based on Improved BP Neural Network

The BP neural network has the following characteristics:

1. The advantage of the neural network is that it has the ability to simulate multiple variables without making complicated correlation assumptions about the input variables
2. One hidden layer is all that is needed to estimate any continuous function on an enclosed area with any degree of accuracy if the number of hidden nodes is enough
3. The generalization ability of BP neural network. After the neural network is trained, it does not respond to small changes in the input, which reflects the inaccuracy of its operation. An inaccuracy is a flaw, yet in certain instances, the system's performance may benefit from it. The purpose of this research is to develop a model for evaluating the quality of teaching by including the BP neural network [20, 21]

The challenge of determining the best model structure design is critical. The number of network trainings may be reduced, and the accuracy of network learning can be improved by making the right decision. This covers the kind of connection, the network level, and how many nodes are in each tier (that is, to determine the number of neurons in the input layer, hidden layer, and output layer). A nonlinear mapping between input (teaching quality evaluation index) and output (final assessment result of instructors' teaching quality) may be used to describe the challenge in teaching quality evaluation. If you want the most accurate approximation possible, a three-layer BP network topology is the best choice for this study.  Figure 3 shows the BP neural network model for the teaching quality evaluation system, which may be summarized as follows. The realization process of the whole system is shown in Figure 4.

## 4. Experiment and Analysis

### 4.1. Determination of the Number of Neurons in Each Layer

Determination of the number of neurons in the input layer: The number of secondary indicators in the theoretical teaching quality evaluation system is 12, so the number of neurons in the input layer is set to 12. In the determination of the number of neurons in the hidden layer: calculated according to the empirical formula, when the initial number of nodes in the hidden layer is 5, multiple network structures are set up, and the number of nodes in the hidden layer of each network is increased by 1. The experimental results are shown in Figure 5; it can be seen that when the number of hidden layer nodes is 5, the error is the smallest, so the number of hidden layer nodes of the BP neural network is set to 5. In the determination of the number of neurons in the output layer, the output target is the teaching quality evaluation result, so the output the layer node is 1.

### 4.2. Preparation and Training of Sample Library

It is critical to have samples accessible when training an artificial neural network. The quality of the sample selection has a direct impact on the neural network's training results. The selection of samples should be based on representative samples based on summing and analysis. Students in the classroom are given a questionnaire based on the teaching quality assessment indicators, which allows them to choose and rate different aspects of their instructors' performance. It is like having a lot of judges in each classroom since there are so many kids. The average value of the instructor's 12 input indications is calculated using the five highest and the five lowest scores, so that certain students' unreliable evaluations of the teacher may be discarded. Rather on relying on a predetermined set of output indicators, this study relies on data from actual classes to train a neural network using evaluations from the teacher oversight group. Although the students write out the teacher's indications, the ultimate assessment outcome reflects the evaluation thoughts of specialists in the supervisory team's group.

The obtained data is standardized using the index system's standardization process. The neural network will be able to handle these data more easily if they are converted to binary data. Tables 2 and 3 show the results of the data processing on the samples. Use the training data in Table 2 and the verification data in Table 3 to check the neural network model's prediction results.

### 4.3. Simulation Experiments and Results

MATLAB's neural network toolbox offers implementations of different neural network algorithm applications. The initialization of a BP neural network for Matlab typically consists of four steps: The establishment of the network is the next step. The third step is a network simulation. The network must be trained as a fourth step. An example of a simulation would be to read in the training data, create an appropriate neural network model using the above-mentioned model structure, and then begin training the model using these parameters. A neural network model is created, validation data is read in, and the predicted value is produced by the network computation when the training is complete.

After the network training, the simulation results were evaluated and the expert results of the five test sets were evaluated (see Figures 6 and 7). All of the training samples were found to be extremely near to expert assessment findings, as shown in Figures 6 and 7, and this was also true for the five simulated test sets. Experimental evidence shows that the BP neural network-based model for evaluating vocational education quality has training and prediction accuracy that is totally acceptable and that the model is a sensible and viable one.

## 5. Conclusion

Because of its great nonlinear learning ability and fault tolerance to noisy input, the BP neural network is the most extensively used artificial neural network method in data mining applications. This paper incorporates the theory of artificial neural networks into the quality evaluation of vocational education and teaching reform, based on extensive research on artificial neural network algorithms. The characteristics of this system are as follows: a comprehensive overview of several commonly used artificial neural network algorithms and a focus on the BP network model structure and learning algorithm; an upgraded version of the BP neural network is proposed in this research to address the issues of poor convergence speed and local minimum points and is used to combine the BP algorithm with the simulated annealing method to form a new algorithm. It can take into account not only the benefits of determining the connection weight adjustment amount in the BP algorithm but also the randomness and heuristics of determining the connection weight adjustment (amount) in the simulated annealing approach. Students of different majors have varied inclinations for different courses because to the randomization of students in the process of evaluating teaching, and due to the involvement of some human variables, students' scores cannot really reflect the actual teaching effect. This study incorporates artificial neural networks into the assessment of teaching quality by utilizing their nonlinear learning ability and fault tolerance. An assessment system for vocational education quality is presented in this research, which shows how the functions of data collecting and evaluation findings may be realized. The teaching quality assessment model built by utilizing neural network gives full play to the benefits of neural network. It is a new way to measure the quality of vocational education.

## Figures and Tables

**Figure 1:** Artificial neuron model.

**Figure 2:** Schematic diagram of three-layer BP neural network structure.

**Figure 3:** BP neural network model for teaching quality assessment.

**Figure 4:** System implementation process.

**Figure 5:** The number of nodes in the hidden layer of the network and the error.

**Figure 6:** Comparison of neural network training results and actual evaluation results.

**Figure 7:** Test set test results compared to actual evaluation.

**Table 1:** Evaluation indicator table.

Indicator category	Label
Rigorous lesson preparation	*X*_1_
Homework correction, tutoring students	*X*_2_
Systemicity of content	*X*_3_
Clearly express complex issues	*X*_4_
Heuristic, auxiliary teaching methods	*X*_5_
Key points, difficult points to deal with	*X*_6_
Motivate students' enthusiasm	*X*_7_
Teaching students according to their aptitude	*X*_8_
Focus on inspiration	*X*_9_
Focus on communicating and interacting with students	*X*_10_
Whether the student's requirements are strict and fair	*X*_11_
Student ability improvement	*X*_12_

**Table 2:** Normalized training data.

Enter	1	2	3	4	5	6	7	8
*X*_1_	0.53	0.64	0.58	0.66	0.96	0.82	0.72	0.59
*X*_2_	0.61	0.53	0.68	0.88	0.73	0.99	0.93	0.59
*X*_3_	0.73	0.61	0.58	0.97	0.85	0.75	0.63	0.67
*X*_4_	0.62	0.85	0.94	0.73	0.59	0.82	0.71	0.66
*X*_5_	0.55	0.97	0.49	0.53	0.84	0.45	0.64	0.77
*X*_6_	0.58	0.99	0.86	0.56	0.78	0.75	0.67	0.54
*X*_7_	0.53	0.64	0.58	0.66	0.96	0.82	0.72	0.59
*X*_8_	0.61	0.53	0.68	0.88	0.73	0.99	0.93	0.59
*X*_9_	0.58	0.99	0.86	0.56	0.78	0.75	0.67	0.54
*X*_10_	0.62	0.85	0.94	0.73	0.59	0.82	0.71	0.66
*X*_11_	0.53	0.64	0.58	0.66	0.96	0.82	0.72	0.59
*X*_12_	0.63	0.71	0.98	0.87	0.75	0.65	0.63	0.65

**Table 3:** Validation data after normalization.

Enter	1	2	3	4	5
*X*_1_	0.55	0.68	0.57	0.58	0.96
*X*_2_	0.66	0.59	0.72	0.88	0.96
*X*_3_	0.78	0.64	0.59	0.96	0.85
*X*_4_	0.58	0.75	0.93	0.65	0.68
*X*_5_	0.59	0.99	0.55	0.67	0.79
*X*_6_	0.57	0.91	0.79	0.82	0.74
*X*_7_	0.65	0.58	0.77	0.98	0.66
*X*_8_	0.76	0.69	0.52	0.98	0.86
*X*_9_	0.68	0.74	0.99	0.56	0.85
*X*_10_	0.78	0.95	0.63	0.75	0.58
*X*_11_	0.89	0.59	0.95	0.77	0.69
*X*_12_	0.67	0.81	0.99	0.72	0.84

## Data Availability

The datasets used during the current study are available from the corresponding author on reasonable request.
